# Shared Genetic and Epigenetic Mechanisms between the Osteogenic Differentiation of Dental Pulp Stem Cells and Bone Marrow Stem Cells

This article has been retracted.

**DOI:** 10.1155/2021/6697810

**Published:** 2021-02-05

**Authors:** Sebastian Gaus, Hanluo Li, Simin Li, Qian Wang, Tina Kottek, Sebastian Hahnel, Xiangqiong Liu, Yupei Deng, Dirk Ziebolz, Rainer Haak, Gerhard Schmalz, Lei Liu, Vuk Savkovic, Bernd Lethaus

**Affiliations:** ^1^Department of Cranio Maxillofacial Surgery, University Clinic Leipzig, Liebigstr. 12, Leipzig 04103, Germany; ^2^Department of Cariology, Endodontology and Periodontology, University Leipzig, Liebigstr. 12, Leipzig 04103, Germany; ^3^Department of Central Laboratory, Taian Central Hospital, Longtan Road No. 29, Taian, 271000 Shandong Province, China; ^4^Department of Molecular Cell Biology, Beijing Tibetan Hospital, China Tibetology Research Center, 218 Anwaixiaoguanbeili Street, Chaoyang, Beijing 100029, China; ^5^Department of Neurology, Shandong Provincial Third Hospital, Cheeloo Chollege of Medicine, Shandong University, Jinan, 100191 Shandong Province, China

## Abstract

**Objective:**

To identify the shared genetic and epigenetic mechanisms between the osteogenic differentiation of dental pulp stem cells (DPSC) and bone marrow stem cells (BMSC).

**Materials and Methods:**

The profiling datasets of miRNA expression in the osteogenic differentiation of mesenchymal stem cells from the dental pulp (DPSC) and bone marrow (BMSC) were searched in the Gene Expression Omnibus (GEO) database. The differential expression analysis was performed to identify differentially expressed miRNAs (DEmiRNAs) dysregulated in DPSC and BMSC osteodifferentiation. The target genes of the DEmiRNAs that were dysregulated in DPSC and BMSC osteodifferentiation were identified, followed by the identification of the signaling pathways and biological processes (BPs) of these target genes. Accordingly, the DEmiRNA-transcription factor (TFs) network and the DEmiRNAs-small molecular drug network involved in the DPSC and BMSC osteodifferentiation were constructed.

**Results:**

16 dysregulated DEmiRNAs were found to be overlapped in the DPSC and BMSC osteodifferentiation, including 8 DEmiRNAs with a common expression pattern (8 upregulated DEmiRNAs (miR-101-3p, miR-143-3p, miR-145-3p/5p, miR-19a-3p, miR-34c-5p, miR-3607-3p, miR-378e, miR-671-3p, and miR-671-5p) and 1 downregulated DEmiRNA (miR-671-3p/5p)), as well as 8 DEmiRNAs with a different expression pattern (i.e., miR-1273g-3p, miR-146a-5p, miR-146b-5p, miR-337-3p, miR-382-3p, miR-4508, miR-4516, and miR-6087). Several signaling pathways (TNF, mTOR, Hippo, neutrophin, and pathways regulating pluripotency of stem cells), transcription factors (RUNX1, FOXA1, HIF1A, and MYC), and small molecule drugs (curcumin, docosahexaenoic acid (DHA), vitamin D3, arsenic trioxide, 5-fluorouracil (5-FU), and naringin) were identified as common regulators of both the DPSC and BMSC osteodifferentiation.

**Conclusion:**

Common genetic and epigenetic mechanisms are involved in the osteodifferentiation of DPSCs and BMSCs.

## 1. Introduction

Repairing bone defects remains a challenge for clinical practitioners to the present day. For the last decades, autologous bone transplantation has been a “gold standard” for treating bone defects in the dental field, such as insufficient bone volume for dental implants and maxillofacial defects [1, 2]. Nonetheless, the conventional treatment involves drawbacks such as donor site morbidity and limitation of bone volume [3], which calls for alternative approaches. Mesenchymal stem cells appear to be a good match to the unmet needs of the conventional autologous bone transplantation. They are capable of acting in paracrine anti-inflammatory and trophic fashion, as well as of providing a cellular base for tissue replacement by virtue of their self-renewal and multilineage differentiation capacity [4]. The most commonly used MSCs are bone marrow stem cells (BMSCs), dental pulp stem cells (DPSCs), and adipose tissue stem cells (ADSCs). BMSCs have been the most commonly used type of stem cells for osteogenesis and new bone formation due to their tissue origin; however, BMSCs are obtained by means of invasive and painful bone marrow aspiration [5]. This downside has inspired the use of other less invasively obtained stem cell types. Among those, DPSCs obtained from the extracted third molar present a highly accessible alternative [6]. In addition, DPSCs have been demonstrated as highly capable of osteogenic differentiation under osteogenesis-inducing conditions [7], and they are therefore becoming a valuable alternative approach for transplantation-based bone regeneration [8]. Nevertheless, critical preclinical data necessary for understanding the genetic and epigenetic mechanisms involved in the osteogenic differentiation of DPSCs and BMSCs are still modestly represented.

Stem cells derived from different tissues tend to respond to the same stimulus differently and differentiate towards the tissue of their origin [9]. Accordingly, BMSCs display a high predisposition to progress towards osteogenic differentiation [9]. It has been shown that the osteogenic differentiation capacity of the BMSCs is higher than that of ADSCs [10, 11] and comparable between the BMSCs and DPSCs [12]. Having tremendous BMSCs and DPSCs osteogenic potential at disposal, it is necessary to gain a fuller understanding of genetic and epigenetic processes that underlie their differentiation capacity in order to utilize their osteogenic ability.

Many genetic and epigenetic factors are involved in the osteogenic differentiation of stem cells, such as messenger RNAs (mRNAs), microRNAs (miRNAs), and signaling pathways. As a significant component of the epigenetic modification, miRNAs are classified as short noncoding RNAs which can inhibit the expression of mRNAs by binding the 3′-untranslated region (UTR) of target mRNAs [13, 14]. The aberrant expression of many miRNAs (e.g., miR-16, miR-381, miR-20a, and miR-214) has been involved in the osteogenic differentiation of stem cells by inducing the dysregulation of osteogenesis-related signaling pathways (e.g., Wnt, BMP, MAPK, RUNX2, and Notch pathways) [15–22]. Although some research using RNA-sequencing technique have investigated the miRNA expression alterations during the osteodifferentiation process of BMSCs [23] and DPSCs [24], respectively, there is still no report which is aimed on identifying the genetic and epigenetic biomarkers shared between the osteogenic differentiation of both types of stem cells.

The present study is aimed at identifying the overlapping genetic and epigenetic mechanisms involved in the osteogenic differentiation of DPSC and BMSC. To this purpose, a series of bioinformatics analyses (e.g., differential expression analysis, DEmiRNA-target gene network construction, DEmiRNA-transcription factor construction, and functional enrichment analysis) were performed to investigate the major common genetic and epigenetic mechanisms of DPSC osteogenesis and BMSC osteogenesis.

## 2. Materials and Methods

### 2.1. Data Acquisition

The miRNA expression profiling datasets regarding the osteogenic differentiation of DPSC and BMSC were searched for in the Gene Expression Omnibus (GEO) database of NCBI [25]. The following inclusion criteria were defined for analyzing two study groups: an undifferentiated control group nominated as the day zero of differentiation (d0), and the experimental group examined after differentiation on day 14, with matched examination days for the DPSC and BMSC experimental group (d14). The datasets with a sample size of more than three for each group were included.

### 2.2. Analyzing Processes of the Present Research

Two datasets (GSE138180 and GSE107279), which investigated the miRNA expression profile of DPSC and BMSC, were selected for assessment. After selecting the corresponding datasets, a series of bioinformatics analyses were performed according to the flowchart of this study (Figure 1).

Firstly, the differential expression analysis was performed to identify the DEmiRNAs which were aberrantly expressed during the osteodifferentiation process of DPSCs and BMSCs, in order to identify the overlapping DEmiRNAs. Subsequently, the target genes of these common DEmiRNAs that were singled out in the first step were identified by constructing a target gene network of 16 overlapping DEmiRNAs. Furthermore, target genes of DEmiRNAs involved in the DPSC osteogenesis and BMSC osteogenesis were, respectively, extracted by searching miRNA-target interaction databases. The functions (i.e., biological processes and signaling pathways) of these target genes were identified by the means of functional enrichment analysis. In addition, transcription factors that potentially target the DEmiRNAs were identified by constructing the DEmiRNAs-transcription factor interaction network. Conclusively, the DEmiRNAs-small molecular drug targets network was constructed in order to identify the small molecular drugs that can influence the expression of DEmiRNAs involved in DPSC and BMSC osteodifferentiation.

### 2.3. Differential Expression Analysis for Identifying DEmiRNAs

Differential expression analysis (DEA) was used to identify the differentially expressed miRNAs (DEmiRNAs) of the two selected datasets. DEA was performed by using different packages in the R program depending on the different experimental types of datasets. The limma package was used to analyze continuous data such as microarray data, whereas the edgeR/DESeq/DESeq2 was used for count data such as high-throughput sequencing. The experimental type of the GSE138180 dataset presents the noncoding RNA profile analyzed by the means of microarray, whereas the experimental type of the GSE107279 dataset profiling of the noncoding RNA has been attained by high-throughput sequencing. Based on this, the DEA of the GSE138180 dataset was carried out using the limma package of the R program version 3.6.1 [26], whereas the DEA of the GSE107279 dataset was performed by using the DESeq2 package [27]. The miRNAs with a *p* value < 0.05 and ∣log FC | ≥1 were selected as differentially expressed. The DEmiRNAs with log FC ≥ 1 was defined as upregulated DEmiRNAs, while the DEmiRNAs with log FC ≤ −1 were defined as downregulated DEmiRNAs. The overlapping DEmiRNAs expressed in the osteogenic differentiation of DPSC and BMSC were found by uploading the list of DEmiRNAs in the Venn web tool webpage (http://bioinformatics.psb.ugent.be/webtools/Venn/).

### 2.4. Target Genes of the Overlapping DEmiRNAs in DPSC and BMSC Osteodifferentiation

After identifying the overlapped DEmiRNAs that were dysregulated in both DPSC and BMSC osteodifferentiation, their target genes were extracted by downloading the human miRNA-target interaction pairs from three databases including miRDB Version 6.0 [28], miRWalk [29], and TargetScan v7.1 [30]. The overlapping DEmiRNA-target gene interaction network was therefore constructed, and the target genes with the top degree were identified.

### 2.5. Functional Enrichment Analysis of Target Genes of DEmiRNAs

After obtaining the DEmiRNAs expressed during the osteogenic differentiation of DPSC and BMSC, target genes of DEmiRNAs involved in DPSC osteodifferentiation and BMSC osteodifferentiation were, respectively, extracted by downloading the human miRNA-target interaction pairs from three databases mentioned earlier [28–30]. The functional enrichment analysis (FEA) was performed on the target genes of DEmiRNAs expressed in the osteogenic differentiation of DPSC and BMSC. This analysis was conducted by using the clusterProfiler package of the R program [31]. The functions of the candidate target genes of the DEmiRNAs were explored by assessing their enrichment in Gene Ontology (GO) terms, in particular biological processes (BPs) and the pathway enrichment analysis according to the Kyoto Encyclopedia of Genes and Genomes (KEGG). The GO terms and KEGG pathways with a *p* value < 0.05 were considered to be significantly enriched. If the number of enriched BPs and pathways was greater than 30, only the top 30 with the highest *p* values were chosen to be visualized in the bar plot. If the number of enriched BPs and pathways was lower than 30, all of the BPs and pathways were visualized in the bar plot.

### 2.6. Construction of DEmiRNA-Transcription Factor (TF) Interaction Network

Based on the DEmiRNAs obtained by DEA, the DEmiRNA-transcription factor (TF) interaction pairs were derived from the TransmiR database [32]. The DEmiRNA-TF regulatory networks involved in the DPSC osteogenesis and BMSC osteogenesis were, respectively, plotted by using the Cytoscape software version 3.7.2. The topological characteristics of the nodes in these two networks were calculated. The top 30 TFs with the highest degree in these two networks were selected, and their intersection was obtained. The intersection between the top 30 TFs of these two networks could be regarded as critical overlapping TFs that targeted DEmiRNAs dysregulated in both the DPSC and BMSC osteodifferentiation.

### 2.7. Construction of DEmiRNA-Small Molecular Drug Target Interaction Network

The SM2miR database provides information about experimentally validated linkage between miRNAs and bioactive small molecules that can influence expression levels of the miRNAs [33]. This database contains 2,925 relationship pairs between small molecule drugs and miRNAs in 17 species, and only the data related to human species were collected. A total of 2,756 human interaction pairs between miRNAs and small molecular drugs were collected from this database. The interaction pairs of (DEmiRNAs (DPSC osteodifferentiation)-small molecule targets) and (DEmiRNAs (BMSC osteodifferentiation)-small molecule targets) were, respectively, extracted from database SM2miR v1.0 [33]. Subsequently, the DEmiRNAs-small molecule drug targets networks were constructed for DPSC and BMSC osteodifferentiation by the means of Cytoscape software version 3.6. In these two networks, the expression patterns (up-/downregulation) of miRNAs were defined according to their expression in the DPSC and BMSC osteodifferentiation, rather than their expression patterns shown in the SM2miR database. Consequently, the intersections between these two networks were identified based on the overlapping DEmiRNA-small molecule interaction pairs and the overlapping small molecules.

## 3. Results

### 3.1. Dataset Procurement

Preselection of data relevant to the miRNA expression profiling of DPSC and BMSC in the course of the osteogenic differentiation process brought about two datasets (GSE138180 and GSE107279). The GSE138180 dataset (https://www.ncbi.nlm.nih.gov/geo/query/acc.cgi?acc= GSE138180) reported the miRNA expression alteration of DPSC investigated by comparing the 14^th^ day of postdifferentiation with the 14^th^ day of culturing cells without differentiation. The GSE107279 dataset (https://www.ncbi.nlm.nih.gov/geo/query/acc.cgi?acc=GSE107279) addressed the miRNA expression alteration of BMSC by comparing the 13^th^ day of postdifferentiation with day 0 (nondifferentiated cells while prior to differentiation).

### 3.2. The Overlapping DEmiRNAs during the Osteogenic Differentiation between DPSC and BMSC

After performing DEA based on two datasets (GSE138180 and GSE107279), 186 DEmiRNAs (122 upregulated and 64 downregulated) and 104 DEmiRNAs (52 upregulated and 52 downregulated) were identified as differentially expressed in the osteogenic differentiation processes of DPSC and BMSC, respectively (Figure 2. File S1 and S2 showed the dysregulation of all DEmiRNAs dysregulated in the osteodifferentiation of DPSCs and BMSCs. The top 30 DEmiRNAs of GSE138180 and GSE107279 were listed in Table 1, ranked in the ascending order of their *p* value. The explanation of the abbreviated parameters shown in Table 1 was listed as below: logFC: log2 fold change; AveExpr: average expression across all samples; *t*: logFC divided by its standard error; *p*.value: raw *p* value (based on *t*) from the test that logFC differs from 0; adj.*p*.Val: Benjamini-Hochberg false discovery rate adjusted *p* value; *B*: log-odds that miRNA is DE; expression patterns: DEmiRNA is upregulated or downregulated.

As shown in the Venn diagram (Figure 2), a total of 186 DEmiRNAs (122 upregulated and 64 downregulated) and 104 DEmiRNAs (52 upregulated and 52 downregulated) were identified to be involved in the osteodifferentiation of DPSCs and BMSCs, respectively. 16 DEmiRNAs were identified as relevant for the osteogenic differentiation of both DPSCs and BMSCs. Among these 16 overlapped DEmiNAs, eight DEmiRNAs (i.e., miR-101-3p, miR-143-3p, miR-145 (3p/5p), miR-19a-3p, miR-34c-5p, miR-3607-3p, miR-378e, and miR-671 (3p/5p)) were found to show the same expression patterns in the osteodifferentiation course (2 weeks) of both DPSCs and BMSCs, while another eight DEmiRNAs (i.e., miR-1273g-3p, miR-146a-5p, miR-4508, miR-4516, miR-6087, miR-146b-5p, miR-337-3p, and miR-382-3p) were found to show the different expression patterns. Among the eight DEmiRNAs with the same expression patterns, seven DEmiRNAs were found to be upregulated in the osteogenic differentiation course (~2 weeks) of both DPSCs and BMSCs: miR-101-3p, miR-143-3p, miR-145(3p/5p), miR-19a-3p, miR-34c-5p, miR-3607-3p, and miR-378e; and another one DEmiRNA (miR-671 (3p/5p)) was found to be downregulated in the osteogenic differentiation course (2 weeks) of both DPSCs and BMSCs. Another eight DEmiRNAs were divergently expressed in DPSCs and BMSCs throughout the osteogenic differentiation course (2 weeks), e.g., five miRNAs were found downregulated in DPSCs while upregulated in BMSCs (i.e., miR-1273g-3p, miR-146a-5p, miR-4508, miR-4516, and miR-6087), as well as three miRNAs upregulated in DPSCs while downregulated in BMSCs (i.e., miR-146b-5p, miR-337-3p, and miR-382-3p). Among these 16 DemiRNAs, 11 of them (i.e., miR-19a-3p, miR-3607-3p, miR-378e, miR-671 (3p/5p), miR-1273g-3p, miR-146b-5p, miR-337-3p, miR-4508, miR-4516, miR-6087, and miR-382-3p) were not supported by previous evidence to be involved in the osteodifferentiation of stem cells. The functions of other five DEmiRNAs (i.e., miR-101-3p, miR-143-3p, miR-145 (3p/5p), miR-34c-5p, and miR-146a-5p) in the osteodifferentiaton of DPSCs and BMSCs were summarized in Table 2.

### 3.3. The Target Genes of the 16 Overlapped DEmiRNAs

In order to identify the target genes of the 16 overlapping DEmiRNAs, their DEmiRNA-target interaction network was constructed (Figure 3). The topological characteristics of all nodes of this network were shown in File S3, and the topological features of the top 30 gene nodes of this network were shown in Table 3. As shown in Table 3, genes CCND2 (cyclin D2), THBS1 (thrombospondin-1), CCND1 (cyclin D1), IGF1R (insulin-like growth factor 1 receptor), REL (REL proto-oncogene, NF-KB subunit), and ELK4 (ETS transcription factor ELK4)) were identified as the target genes of 16 DEmiRNAs.

### 3.4. The Overlapping Biological Processes and Pathways Involved in the Osteogenic Differentiation of DPSCs and BMSCs

Subsequently, by the means of the functional enrichment analysis, the significantly enriched biological processes (BPs) and signaling pathways in target genes of the DEmiRNAs were identified for DPSCs and BMSCs (Figures 4 and 5). The overlapping BPs and pathways involved in the osteogenic differentiation of DPSCs and BMSCs were singled out. As shown in Figure 4, several BPs were identified as overlapping and therefore common for osteogenic differentiation of both DPSCs and BMSCs: p53 binding, protein heterodimerization activity, ATPase activity, GTPase binding, cadherin binding, and histone binding DPSCs and BMSCs. As shown in Figure 5, a total of 12 signaling pathways were identified as overlapped between DPSCs and BMSCs: TNF, mTOR, Hippo, neutrophin, pathways regulating pluripotency of stem cells, cell cycle, MAPK, focal adhesion, ubiquitin-mediated proteolysis, viral carcinogenesis, autophagy, and protein processing in endoplasmic reticulum and endocytosis.

### 3.5. The Overlapping Transcription Factors Targeted by DEmiRNAs between DPSCs and BMSCs

As shown in Figure 6, the DEmiRNA-transcription factor (TF) interaction network involved in both DPSCs and BMSCs were constructed. The top 30 TFs with the highest degree in these two networks were listed in Table 4 ranking in the descending order of degree. By comparing the top 30 TFs with the highest degree in these two networks shown in File S4 and File S5, a total of 26 transcription factors were found overlapped, e.g., TCF12, ERG, CEBPB, ELF1, TCF3, ARNTL, KDM2B, MYC, BRD4, CTCF, MAX, LARP7, HIF1A, E2F1, KDM5B, MAZ, PHF8, STAT1, EP300, AR, FOXA1, TFAP2C, RUNX1, ESR1, TRIM28, and SPI1.

### 3.6. The Overlapping Small Molecules Targeted by DEmiRNAs Dysregulated in DPSCs and BMSCs Osteodifferentiation

The DEmiRNA-small molecular drug target interaction network, respectively, involved in DPSCs and BMSCs osteodifferentiation were shown in Figures 7(a) and 6(b). In the SM2miR database, only 40 DEmiRNAs of DPSC osteodifferentiation and 27 DEmiRNAs of BMSC osteodifferentiation were found to be targeted and regulated by the small molecular drugs. The small molecular drugs in this database were not found to target and impact the expression of the other DEmiRNAs that were also dysregulated in DPSC and BMSC osteodifferentiation. By assessing the interaction pairs shown in Figures 7(a) and 7(b), we identified 13 interaction pairs consisting of four DEmiRNAs (hsa-miR-143-3p, hsa-miR-146b-5p, hsa-miR-34c-5p, and hsa-miR-671-5p). 13 small molecules were found to be shared between the two networks that are displayed in Table 5. Additionally, a total of 19 small molecule drugs were found to not only impact the expression of DEmiRNAs in DPSC osteodifferentiation but also that of DEmiRNAs in BMSC osteodifferentiation: 5-fluorouracil, anthocyanin, arsenic trioxide, ascorbate, atorvastatin, bromocriptine, curcumin, docosahexaenoic acid, ginsenoside Rh2, glucose, hesperidin, hydroxycamptothecin (HCPT), microcystin-LR (MC-LR), mistletoe lectin-I, narangin, proanthocyanin, progesterone, vitamin D3, and vorinostat (SAHA).  Table 6 shows the targeting relationship between 19 overlapping small molecule drugs and their regulated DEmiRNAs, respectively, expressed in DPSC and BMSC osteodifferentiation process.

## 4. Discussion

This study identifies multiple genetic and epigenetic biomarkers common for osteogenic differentiation of DPSCs and BMSCs, including miRNAs, their target genes, transcription factors, signaling pathways, and small molecular drugs affecting those mentioned. The overlapping miRNAs with the same expression pattern in DPSC and BMSC osteodifferentiation were obtained by investigating the dysregulated DEmiRNAs in both DPSC and BMSC osteogenesis. The target genes of those shared DEmiRNAs were identified by constructing the shared DEmiRNA-target gene network. The TFs among those genes, signaling pathways involved, and small molecule drugs that predictively affect those pathways were identified as highly plausible common regulators of the osteodifferentiation process in both DPSCs and BMSCs. Their involvement in DPSC and BMSC osteodifferentiation will be discussed here.

This discussion addresses several of the eight miRNAs that were found to be differentially expressed, with the same expression pattern in the course of osteogenic differentiation of DPSCs and BMSCs (miR-101-3p, miR-143-3p, miR-145 (-3p/-5p), miR-19a-3p, miR-34c-5p, miR-3607-3p, miR-378e, and miR-671 (-3p/-5p)). Since there has not been any evidence showing the involvement of miR-19a, miR-3607, miR-378e, and miR-671 in osteogenesis of stem cells, we excluded them from further discussion in order to avoid speculation. The possible role of the other four miRNAs (miR-101, miR-143, miR-145, and miR-34 family (miR-34a/b/c)) will be interpreted in the following part of this section. Overexpression of miR-101 was shown to target EZH2/Wnt/*β*-Catenin signaling, hereby promoting the osteogenic differentiation in general [34]. Nevertheless, no evidence has been produced to corroborate the expression pattern and either promoting or an inhibiting role of miR-101 during the osteogenesis of DPSCs. The miR-143 has been designated with an evident inhibiting role in osteogenesis and odontogenesis. Downregulation of miR-143 has been shown to promote the osteogenic and odontogenic differentiation of DPSCs by activating the NF-*κ*B [36] and OPG/RANKL signaling [37]. The decreased expression of miR-143 was also shown to promote the osteogenic differentiation of BMSCs by being competitively combined with lncRNA MALAT1 and further upregulating the expression of Osterix (Osx), suggesting that MALAT1-miR-143-Osx could be an integrative element in the ceRNA network of BMSC osteogenesis [35]. Opposite to the results shown in these previous studies, the present study shows an upregulation of miR-143 during the osteogenic differentiation in both BMSCs and DPSCs. miR-145 (-3p/-5p) appears to function the same way as miR-143. The downregulation of miR-145 can apparently promote the odontoblast differentiation of DPSC by targeting transcriptional factor KLF4 and OSX [39]. Also, the downregulation of miR-145 can promote osteogenic differentiation of BMSC by targeting semaphorin3A (SEMA3A), a known positive regulator of osteogenesis [38]. Similarly to the miR-143, the expression pattern of miR-145 shown in the previous work of others is not in agreement with the *in silico* data derived from the datasets analyzed in this study, which show that miR-145 is overexpressed in the course of osteodifferentiation of both DPSCs and BMSCs. The miR-34 family (miR-34a/b/c) has so far not been designated as categorically pro- or counterosteogenic in DPSCs. Two surveys have shown the involvement of the miR-34 family in the osteogenic differentiation of BMSC [43, 44], however, with quite contradictory results about its expression pattern. Chen et al. showed that miR-34a could inhibit osteogenesis by suppressing regulators cell cycle and cell proliferation cyclin D1, CDK4, and CDK6 [43] and that the inhibition of miR-34a could facilitate osteogenesis of BMSCs. Contrary to that, Xin et al. showed that the upregulation of miR-34a could promote osteogenesis of BMSCs and reverse proinflammatory cytokine influence by targeting tumor necrosis factor-alpha (TNF-*α*) [45]. Altogether, the osteogenesis-relevant DEmiRNAs that were found overlapping in DPSCs and BMSCs are involved in signaling pathways that regulate differentiation and inflammatory processes by targeting their major regulators.

After identifying 16 overlapping DEmiRNAs, the target genes of these 16 DEmiRNAs were also identified by constructing the corresponding DEmiRNA-target gene network. Among the top 30 target genes of 16 overlapping DEmiRNAs, only some typical examples of genes will be discussed based on the previous literature evidence regarding their involvement in the osteodifferentiation of DPSCs and BMSCs (e.g., REL, CCND1/2, IGF1R, THBS1, and ELK4). REL gene family consists of RelA (p65), RelB, and c-Rel, subunits of NF-KB. Activation of NF-KB subunit RelA (p65) was shown to significantly promote inflammation and inhibit osteodifferentiation of BMSCs by promoting the ubiquitination and degradation of beta-catenin, indicating that inhibitors of RelA (p65) could be a novel therapeutic target for inhibiting inflammation and enhancing osteogenesis [46]. In accordance with the findings shown in BMSCs, studies investigating DPSCs also showed that the downregulation of NF-KB subunit RelA (p65) enhanced the odontogenic/osteogenic differentiation of DPSCs [47, 48]. Cyclin D genes are involved in cell cycle regulation. Silencing of cyclin D genes (CCND1/2) was shown to arrest the cell cycle, and its overexpression has been connected to the progression of the cell cycle [49]. That the data regarding the effects of cell cycle regulators on osteodifferentiation have so far been insufficiently coherent, CCND1/2 expression was significantly upregulated in the course of DPSC osteodifferentiation [50, 51], whereas during BMSC differentiation the genes involved in the cell cycle were significantly downregulated [52]. IGF1R (insulin-like growth factor 1 receptor) can bind IGF1 with a high affinity [53]. The previous studies regarding BMSCs also showed that IGF1 promoted osteodifferentiation of BMSCs and could even be regarded as an alternative biomarker to bone morphogenetic protein-7 [54, 55]. In addition, the IGF axis (e.g., IGF-2 and IGFBP-2) was activated under osteogenic conditions in DPSCs, indicating its promoting role in DPSC osteodifferentiation [56]. THBS1 (thrombospondin-1) is a major regulator of latent TGF-*β* activation [57], which can inhibit osteoblast differentiation in BMSCs. Accordingly, THBS1 was found to inhibit the osteodifferentiation of BMSCs by activating the TGF-*β* pathway [58]. An analogue involvement of THBS1 in osteodifferentiation of DPSCs has not been reported yet. Another modulator of osteogenic differentiation ELK4 (ETS transcription factor ELK4) was also predicted to be among the target genes of 16 DEmiRNAs. Ets trasnscription factor consisting of Ets1 and Ets2 targets several osteogenic markers (e.g., osteocalcin, osteopontin, bone sialoprotein, and osteonectin) in BMSCs [59]. However, the evidence regarding the regulation of Ets transcription factor in the osteodifferentiation of DPSC is still lacking and thus could be a novel topic for future research.

Among the 13 transcription factors found to be overlapped between the top nodes of the DPSC and BMSC osteogenesis DEmiRNA-TF network, four TFs (RUNX1, FOXA1, HIF1A, and MYC) have been reported relevant for osteodifferentiation of stem cells. Upregulation of Runt-related transcription factor 1 (RUNX1) was shown to promote osteogenesis of BMSCs by activating the canonical Wnt/*β*-catenin pathway [60]. RUNX1 involvement in DPSC osteogenesis has not been shown; nevertheless, another member of the RUNX family (RUNX2) could enhance bone deposition and facilitate novel bone formation after transplantation of RUNX2-transfected DPSCs [61]. Forkhead box protein A1/2 (FOXA1/2) has been reported as hypermethylated in the course of BMSC osteogenesis [62] and its knockdown promoted BMSC osteodifferentiation [63], which has still not been reported in DPSCs. Hypoxic conditions are known to promote cell proliferation and enhance the osteogenic differentiation of both BMSC and DPSC by inducing the expression of HIF1A (hypoxia-inducible factor 1-alpha) and upregulating the osteogenic-related genes (e.g., Oct-4, Sox2, c-Myc, RUNX2, and PPAR*γ*2) [64–66]. HIF1A overexpression in BMSC can induce the overexpression of proosteogenic genes and enhance the ALP activity even in normoxic conditions [67]. However, there is still no direct evidence on the regulating role of HIF1A in the osteodifferentiation process of DPSC. Overexpressed c-MYC was mainly shown to inhibit osteogenic differentiation of both BMSC [68] and DPSC [69]. In DPSCs, stably expressed c-MYC inhibited cell growth during osteogenic differentiation and also impaired the osteogenic phenotypes (i.e., ALP activity and expression of osteogenic marker genes) [69]. On the other hand, a microarray study of gene expression in BMSCs indicated that c-MYC mediated an upregulation of dexamethasone (DEX) expression and of the bone morphogenetic protein 2- (BMP2-) induced osteoblast differentiation [70]. Involvement of other overlapping TFs (e.g., CTCF, BRD4, MAX, ERG, KDM5B, MAZ, EP300, AR, and ESR1) in the osteogenic differentiation of BMSC and DPSC has not been reported yet; thus, these TFs could present novel investigating markers for future research.

A total of 12 overlapping signaling pathways were found to be enriched by the target genes of DEmiRNAs that are involved in the DPSC osteogenesis and BMSC osteogenesis. Among these 12 signaling pathways, five were selected as highly relevant (i.e., TNF, mTOR, Hippo, neutrophin, and signaling pathways regulating pluripotency of stem cells), as the most thoroughly researched and recognized as classic pathways in the osteogenesis of stem cells. Tumor necrosis factor (TNF) signaling cascade has been shown to affect osteogenic differentiation in DPSCs in a dose-dependent manner: proosteogenic at lower doses via activating NF-*κ*B signaling pathway [71] and osteosuppressing at higher doses by modulating the Wnt/*β*-catenin signaling [72]. In BMSCs, the osteosuppressing effect of TNF-*α* is exerted through the downregulation of miR-34a and miR-21 expression [73], which are listed among the top 30 dysregulated DEmiRNAs in osteodifferentiation of BMSCs. The mTOR signaling pathway is activated by stimulation with dexamethasone and kaempferol in DPSCs and BMSCs, respectively, suggesting mTOR as a common pathway in the course of their osteogenesis [74, 75]. Hippo signaling pathway promotes osteogenic differentiation in DPSCs upon regulation by SOX2 and the downstream BMP signaling [76]. In murine BMSCs, the activation of this pathway was induced by calcitonin gene-related peptide (CGRP) and it promoted osteogenic differentiation. Neurotrophin-mediated signaling pathway with rain-derived neurotrophic factor (BDNF) as a key mediator is primarily active in neurogenesis [77] but also intensively involved in osteogenesis of both DPSCs and BMSCs. In DPSCs, the upregulation of BDNF was shown to promote the odontogenic differentiation of DPSCs towards odontoblast-like cells [78] and to indirectly promote osteogenesis in BMSCs [79]. In addition, a plethora of signaling pathways that regulate the pluripotency of stem cells provides the basic framework for any differentiation, including the endpoint bone. Among several key mediators, transforming growth factor-beta (TGF-*β*) signaling is of particular importance, being implicated in regulatory pathways relevant for osteodifferentiation as well. The activation of the TGF-*β* pathway promotes osteogenesis in DPSCs by upregulating osteoblast marker genes type I collagen, alkaline phosphatase (ALP), osteocalcin (OCN), and RUNX2 [80], whereas in BMSCs, its function regarding osteogenesis has been reported in controversial contexts [81, 82].

Apart from the genetic and epigenetic biomarkers, this research also identified 19 small molecular drugs with a simultaneous predictive impact on the DEmiRNAs that are dysregulated in both DPSC and BMSC osteodifferentiation. This section will focus on several of those small molecules that exhibit clear anti-inflammatory or proosteogenic effect in BMSCs: curcumin, docosahexaenoic acid (DHA), vitamin D3, arsenic trioxide, 5-fluorouracil (5-FU), and naringin. Curcumin, a natural phenolic biphenyl compound derived from the plant Curcuma longa, is an antioxidant with anti-inflammatory and osteogenesis-regulating effects [83, 84]. In BMSCs, curcumin facilitates differentiation towards osteoblasts by activating Akt/GSK3*β* and Wnt/*β*-catenin pathways [85]. Docosahexaenoic acid (DHA) belongs to the omega-3 polyunsaturated fatty acids, and it is well-known for being protective against inflammation. DHA promotes the osteodifferentiation of BMSCs by leading to the upregulation of proosteogenic proteins bone-sialoprotein 2 (BSP2), ALP, and RUNX2 [86]. The 1*α*,25-dihydroxyvitamin D_3_, an active metabolite of vitamin D, is crucial for the maintenance of calcium homeostasis and balance of bone remodeling. It induces differentiation of human BMSCs and dental bud stem cells (DBSCs) towards osteoblasts by increasing the expression levels of osteogenic markers (RUNX2, collagen I (Coll I), ALP, osteopontin, and osteocalcin) [87, 88]. Arsenic trioxide (ATO) is a drug which has been commonly used in treating acute promyeloid leukemia (APL) [89]. Additionally, ATO was shown to promote the osteogenic differentiation of BMSC while inhibiting their adipogenic differentiation [90, 91]. The 5-fluorouracil (5-FU) is a commonly used drug in cancer treatment based on inducing the cell death of cycling cells [92]. BMSCs treated with 5-FU exhibited an enhanced osteodifferentiation [93]. Naringin is a dihydrotestosterone flavonoid compound known to promote osteodifferentiation of BMSCs by downregulating expression levels of peroxisome proliferator-activated receptor *γ* (PPAR*γ*) [94]. It has still not been demonstrated if the proosteogenic or anti-inflammatory effects of the mentioned small molecular drugs found in BMSCs exert the same impact in DPSCs. Nevertheless, since the selection of candidates is a result of multiply derived and highly overlapping calculations and predictions employed in this study, we are leaving room for a confident extrapolation of the drug effects on the DPSCs as well.

Apart from discussing the main outcomes, it is noteworthy to mention the limitations of this study. Although mRNA and lncRNA expression profiles related to the osteodifferentiation of DPSCs and BMSCs were available in public databases, they were not included in the analysis. Undoubtedly useful raw data from these datasets did not apply to the common differentially expressed miRNAs in DPSC and BMSC osteodifferentiation. Also, analyzing mRNA and lncRNA expression profiles would have required an entirely different, amiss the scope of the intended study.

The study design of the two analyzed datasets varied in terms of experimental conditions. The experimental group used to generate that the GSE138180 dataset was treated by odontogenic differentiation medium, whereas the control group was cultured in the nondifferentiating medium for two weeks. Even though the DPSCs in control were not stimulated to differentiate and they were therefore regarded as naive in the original study that generated GSE138180, the culturing conditions may have still left room for spontaneous differentiation [24]. The authors interpreted the absence of mineral nodes in the control group, which is a standard sign of the absence of osteogenic differentiation, as an absence of spontaneous differentiation altogether. By all means, this presents sufficient evidence that no osteodifferentiation took place in the control group [24]. Nevertheless, BMSCs can spontaneously differentiate to osteoblasts [95], which imposes a question if the DPSCs can do it too. The experimental design of the study generated the GSE107279 compared the two weeks of post-differentiation with day 0, hereby ensuring that the control group did not spontaneously differentiate. Hereby, the control groups in the two datasets ‘nondifferentiated while not stimulated' in GSE138180 and ‘nondifferentiated while prior to differentiation' in GSE107279 were compared as peer groups. In the lack of further osteogenesis-relevant datasets for BMSCs and DPSCs and considering the argument on the nondifferentiated control group provided by the authors of GSE138180, we carried out the comparative analysis of the two mentioned datasets. Optimally though, experimental set up should be established with a control group at d0 (without culturing and prior to any differentiation) and the experimental group on d14 (after culturing in the osteodifferentiation medium).

In addition, it is important to mention that the osteogenic induction media (50 mg/mL ascorbic acid, 100 nmol/L dexamethasone, and 10 mmol/L *β*-glycerolphosphate) used for GSE138180 could either induce DPSCs towards the osteogenic differentiation and form osteoblasts, or towards the odontogenic differentiation, hereby forming odontoblasts. The authors of GSE138180 regarded the odontogenic and osteogenic differentiation as the same process and reported an odontogenic differentiation of DPSCs in their publication [24] and osteogenic differentiation in the resulting GEO dataset summary (https://www.ncbi.nlm.nih.gov/geo/query/acc.cgi?acc=GSE138180). In the future, potential confusion in investigating the osteogenic/odontogenic differentiation could easily be resolved by assessing odontogenic biomarkers such as dentin matrix acid phosphoprotein 1 (DMP1), dentin sialophosphoprotein (DSPP), and matrix extracellular phosphoglycoprotein (MEPE) [96]. To this day, much of the interpretation of previous work has been limited by not assessing those differential markers [97–102]. Except for this difference, the genetic and epigenetic mechanisms involved in the osteodifferentiation and odontodifferentiation of DPSCs are common [96]. For the purpose of this study, we adopted the reported statement that DPSCs underwent osteogenic differentiation that was comparable to the osteogenic differentiation of BMSCs.

Availibility of only one time point—2 weeks of osteodifferentiation—for analysis of the DPSC-endpoint-bone in GSE138180 presents another limitation in assessing the gradual process of differentiation. Assessing genetic and epigenetic status over several time points could be crucial for understanding the DPSC differentiation dynamics [103]. Analyzing further data points of the DPSC osteodifferentiation could be extremely helpful for their comparison with the already available multiple time points of the BMSC osteodifferentiation.

Last but not least, this study presents computational predictions based on the reported existing raw data. The predictive data have not been directly experimentally validated. Further validation of the biomarkers predicted in this research could be performed by polymerase chain reaction (PCR) and western blotting assays. Despite the stated limitations, the biomarkers identified in the study provide potential directions for future surveys of genetic and epigenetic biomarkers as well as regulatory mediators involved in osteogenic differentiation of DPSCs.

Eventually, the DPSCs and BMSCs appear to share common DEmiRNAs and their targets, with cohesive outcomes on the genetic and epigenetic levels in terms of the osteodifferentiation process. This places them among common targets that could be directly or indirectly influenced by the mentioned selected small molecule drug candidates. The established correlations provide a base for a better understanding of the common molecular alterations during the osteogenic differentiation of DPSCs and BMSCs. Those could present an immense potential if used for tissue engineering purposes, especially drug delivery, herewith putatively contributing to the future therapeutical trends in bone regeneration.

## 5. Conclusions

Several miRNAs (miR-101-3p, miR-143-3p, miR-145-3p, miR-145-5p, miR-19a-3p, miR-34c-5p, miR-3607-3p, miR-378e, miR-671-3p, and miR-671-5p, miR-671-3p, and miR-671-5p), genes (REL, CCND1/2, IGF1R, THBS1, and ELK4), signaling pathways (TNF, mTOR, Hippo, neutrophin, and signaling pathways regulating pluripotency of stem cells), transcription factors (RUNX1, FOXA1, HIF1A, and MYC), and small molecular drugs (curcumin, docosahexaenoic acid (DHA), vitamin D3, arsenic trioxide, 5-fluorouracil (5-FU), and naringin) emerged as shared regulating factors during the osteogenic differentiation of DPSCs and BMSCs. The biomarkers and small molecular drugs identified in this study could be used for the genetic/epigenetic manipulation and drug delivery of DPSCs and therefore result in novel strategies for bone tissue engineering.

## Figures and Tables

**Figure 1:** The study flowchart.

**Figure 2:** 16 DEmiRNAs identified to be overlapped in the osteodifferentiation of DPSCs and BMSCs.

**Figure 3:** The overlapping 16 DEmiRNA-target gene network. The top 30 target genes with the highest degree were displayed enlarged in the network.

**Figure 4:** The enriched biological processes involved in the osteogenic differentiation of DPSC (a) and BMSC (b).

**Figure 5:** The enriched signaling pathway involved in the osteogenic differentiation of DPSC (a) and BMSC (b).

**Figure 6:** The DEmiRNA-TF interaction network involved in the osteogenic differentiation of DPSC (a) and BMSC (b).

**Figure 7:** The DEmiRNA-small molecular drug targets the interaction network involved in the osteogenic differentiation of DPSC (a) and BMSC (b).

**Table 1:** The top 30 DEmiRNAs expressed in the osteogenic differentiation of DPSCs and BMSCs, ranked in the ascending order of their *p* value.

The top 30 DEmiRNAs dysregulated in DPSC osteodifferentiation				
DEmiRNAs	logFC	*p*.value	Adj.*p*.Val	Expression pattern
hsa-let-7f-2-3p	4.542015233	1.45*E* − 06	0.000106517	Up
hsa-miR-1468-3p	4.542015233	1.45*E* − 06	0.000106517	Up
hsa-miR-153-3p	4.542015233	1.45*E* − 06	0.000106517	Up
hsa-miR-212-5p	4.542015233	1.45*E* − 06	0.000106517	Up
hsa-miR-2355-5p	4.542015233	1.45*E* − 06	0.000106517	Up
hsa-miR-342-5p	4.542015233	1.45*E* − 06	0.000106517	Up
hsa-miR-3658	4.542015233	1.45*E* − 06	0.000106517	Up
hsa-miR-450a-1-3p	4.542015233	1.45*E* − 06	0.000106517	Up
hsa-miR-450b-3p	4.542015233	1.45*E* − 06	0.000106517	Up
hsa-miR-4639-5p	4.542015233	1.45*E* − 06	0.000106517	Up
hsa-miR-4730	4.542015233	1.45*E* − 06	0.000106517	Up
hsa-miR-508-3p	4.542015233	1.45*E* − 06	0.000106517	Up
hsa-miR-548d-5p	4.542015233	1.45*E* − 06	0.000106517	Up
hsa-miR-588	4.542015233	1.45*E* − 06	0.000106517	Up
hsa-miR-6077	4.542015233	1.45*E* − 06	0.000106517	Up
hsa-miR-99a-3p	4.542015233	1.45*E* − 06	0.000106517	Up
hsa-miR-1203	4.1591475	2.09*E* − 06	0.000106517	Up
hsa-miR-1238-5p	4.1591475	2.09*E* − 06	0.000106517	Up
hsa-miR-128-2-5p	4.1591475	2.09*E* − 06	0.000106517	Up
hsa-miR-1288-5p	4.1591475	2.09*E* − 06	0.000106517	Up
hsa-miR-129-5p	4.1591475	2.09*E* − 06	0.000106517	Up
hsa-miR-138-1-3p	4.1591475	2.09*E* − 06	0.000106517	Up
hsa-miR-141-3p	4.1591475	2.09*E* − 06	0.000106517	Up
hsa-miR-1972	4.1591475	2.09*E* − 06	0.000106517	Up
hsa-miR-3074-5p	4.1591475	2.09*E* − 06	0.000106517	Up
hsa-miR-339-5p	4.1591475	2.09*E* − 06	0.000106517	Up
hsa-miR-33a-3p	4.1591475	2.09*E* − 06	0.000106517	Up
hsa-miR-34b-3p	4.1591475	2.09*E* − 06	0.000106517	Up
hsa-miR-369-3p	4.1591475	2.09*E* − 06	0.000106517	Up
hsa-miR-382-3p	4.1591475	2.09*E* − 06	0.000106517	Up
The top 30 DEmiRNAs dysregulated in BMSC osteodifferentiation				
DEmiRNAs	logFC	*p*.value	Adj.*p*.Val	Expression pattern
hsa-miR-3182	-5.37979	5.96*E* − 105	3.54*E* − 102	Up
hsa-miR-182-5p	2.561101	1.58*E* − 69	4.67*E* − 67	Down
hsa-miR-335-3p	5.160868	3.61*E* − 59	7.13*E* − 57	Down
hsa-miR-4284	-5.15177	2.73*E* − 56	4.05*E* − 54	Up
hsa-miR-92b-3p	1.590835	1.49*E* − 45	1.76*E* − 43	Down
hsa-miR-21-5p	-1.35202	5.02*E* − 44	4.96*E* − 42	Up
hsa-miR-101-3p	-1.49927	2.63*E* − 43	2.23*E* − 41	Up
hsa-miR-181a-5p	-1.3232	2.30*E* − 37	1.70*E* − 35	Up
hsa-miR-143-3p	-1.96642	1.91*E* − 34	1.26*E* − 32	Up
hsa-miR-210	2.509065	8.42*E* − 34	4.99*E* − 32	Down
hsa-miR-146a-5p	-3.4374	1.93*E* − 33	1.04*E* − 31	Up
hsa-miR-192-5p	-1.78251	2.03*E* − 31	1.00*E* − 29	Up
hsa-miR-146b-5p	2.019632	4.61*E* − 30	2.10*E* − 28	Down
hsa-miR-335-5p	4.772695	3.12*E* − 28	1.32*E* − 26	Down
hsa-miR-382-5p	2.241351	1.20*E* − 25	4.76*E* − 24	Down
hsa-miR-4485	-6.6002	4.46*E* − 24	1.65*E* − 22	Up
hsa-miR-27b-5p	1.588671	2.77*E* − 21	9.68*E* − 20	Down
hsa-miR-10b-5p	-1.21399	4.59*E* − 20	1.51*E* − 18	Up
hsa-miR-4532	-6.35341	5.95*E* − 19	1.86*E* − 17	Up
hsa-miR-34c-5p	-1.82262	8.35*E* − 18	2.36*E* − 16	Up
hsa-miR-181c-5p	-1.15476	1.18*E* − 17	3.19*E* − 16	Up
hsa-miR-409-3p	1.1162	1.06*E* − 15	2.73*E* − 14	Down
hsa-miR-218-5p	1.374343	2.30*E* − 15	5.61*E* − 14	Down
hsa-miR-22-5p	2.004899	2.36*E* − 15	5.61*E* − 14	Down
hsa-miR-133b	-6.46427	4.93*E* − 14	1.08*E* − 12	Up
hsa-miR-3195	-5.55444	5.12*E* − 14	1.09*E* − 12	Up
hsa-miR-133a	-6.42493	6.09*E* − 14	1.24*E* − 12	Up
hsa-miR-6723-5p	-3.89682	7.78*E* − 12	1.44*E* − 10	Up
hsa-miR-4497	-3.78672	1.67*E* − 11	3.00*E* − 10	Up
hsa-miR-4488	-7.47261	2.43*E* − 11	4.11*E* − 10	Up

**Table 2:** The dysregulation and function of five overlapping DEmiRNAs (miR-101-3p, miR-143-3p, miR-145 (3p/5p), miR-34c-5p, and miR-146a-5p) in the osteodifferentiation of BMSCs and DPSCs, respectively.

	BMSC osteodifferentiation	DPSC osteodifferentiation
miR-101-3p	The overexpression of miR-101 promoted the osteogenic differentiation of BMSCs by targeting EZH2/Wnt/*β*-catenin signaling [34].	No evidence.
miR-143-3p	The downregulation of miR-143 promoted the osteogenic differentiation of BMSCs by being competitively combined with lncRNA MALAT1 and upregulating Osterix (Osx) [35].	The downregulation of miR-143 promoted the osteogenic differentiation of DPSCs by activating the NF-*κ*B [36] and OPG/RANKL signaling [37].
miR-145 (3p/5p)	The downregulation of miR-145 promoted the osteogenic differentiation of BMSCs by targeting semaphorin3A (SEMA3A) [38].	The downregulation of miR-145 promoted the odontoblast differentiation of DPSCs by targeting KLF4 and OSX [39].
miR-34c-5p	The upregulation of miR-34c inhibited osteoblast differentiation of BMSCs by targeting the Notch signaling [40].	No evidence.
miR-146a-5p	The overexpression of miR-146a inhibited the osteogenic ability of BMSCs by targeting Smad4 gene [41].	The overexpression of miR-146a-5p promoted osteodifferentiation of DPSCs by suppressing Notch signaling [42].

**Table 3:** The topological characteristics of the top 30 target genes with the highest degree in the 16 overlapping DEmiRNA-target gene network. Typically, this table would be displaying only the top 30 target genes with the highest degree; since 26 target genes were ranked with the degree of 6, a total of 39 target genes with a degree ≥ 6 were finally listed in this table.

Name	Degree	Average shortest path length	Betweenness centrality	Closeness centrality	Topological coefficient
BTG2	8	2.431705	0.003363	0.411234	0.18598065
CCND2	8	2.517604	0.003716	0.397203	0.16845654
NUFIP2	8	2.449032	0.003768	0.408325	0.18394988
THBS1	8	2.231521	0.005344	0.448125	0.17855649
UBN2	8	2.587281	0.004042	0.386506	0.17526212
GIGYF1	8	2.589493	0.003609	0.386176	0.17635862
CCND1	7	2.485899	0.002815	0.402269	0.19450361
IGF1R	7	2.426175	0.003724	0.412171	0.19710456
IREB2	7	2.631152	0.00312	0.380062	0.20047142
REL	7	2.838341	0.002574	0.352318	0.19393939
TNRC6A	7	2.514286	0.002822	0.397727	0.20702541
UHMK1	7	2.499171	0.002866	0.400133	0.20764488
MDM2	7	2.519816	0.003737	0.396854	0.19915693
ADAM10	6	2.52682	0.001899	0.395754	0.24168969
CDKN1A	6	2.667281	0.001979	0.374914	0.2337037
EIF4G2	6	2.655853	0.001796	0.376527	0.23616084
ELK4	6	2.542304	0.001911	0.393344	0.24100872
ETNK1	6	2.726636	0.001859	0.366752	0.23112339
HNRNPU	6	2.652903	0.001945	0.376946	0.23472566
HNRNPUL1	6	2.610876	0.001817	0.383013	0.23927525
LRRC58	6	2.652903	0.001945	0.376946	0.23472566
MAP1B	6	2.741382	0.001822	0.364779	0.21069923
NACC1	6	2.780092	0.002673	0.3597	0.22723133
PANK3	6	2.901382	0.002215	0.344663	0.20067454
PRDM2	6	2.437235	0.002245	0.410301	0.22983744
PURB	6	2.785622	0.002027	0.358986	0.2084477
REV3L	6	2.652166	0.001623	0.37705	0.23674815
RREB1	6	2.823594	0.002115	0.354159	0.20654912
SFT2D2	6	2.652166	0.001623	0.37705	0.23674815
TET3	6	2.52682	0.001899	0.395754	0.24168969
TMBIM6	6	2.52682	0.001899	0.395754	0.24168969
TNPO1	6	2.567373	0.002674	0.389503	0.23314389
ZNF264	6	2.627834	0.001775	0.380542	0.23815304
ZNF678	6	2.57106	0.001949	0.388945	0.23931624
ALDOA	6	2.781198	0.002859	0.359557	0.21913299
CCDC80	6	2.662488	0.00286	0.375588	0.20698404
NF2	6	3.205161	0.002464	0.311997	0.2200685
CBX6	6	2.693456	0.001811	0.37127	0.2316048
DDX21	6	2.772719	0.001683	0.360657	0.22691611

**Table 4:** DEmiRNA-transcription factor (TF) interaction network involved in DPSC and BMSC osteodifferentiation. The top 30 TFs with the highest degree of difference in the DEmiRNA-TF network of DPSCS and BMSCS osteodifferentiation were, respectively, ranked in the descending order of degree.

The top 30 TFs with the highest degree in DEmiRNAs-TF network of DPSC osteodifferentiation					
Name	Degree	Average shortest path length	Betweenness centrality	Closeness centrality	Topological coefficient
FOXA1	30	1.954545	0.015768	0.511628	0.223996
BRD4	29	2.008021	0.009367	0.498003	0.244796
AR	29	2.029412	0.012695	0.492754	0.226894
MAX	29	1.997326	0.009458	0.500669	0.245836
EP300	28	1.981283	0.010644	0.504723	0.248155
ESR1	27	2.024064	0.01016	0.494055	0.226708
HIF1A	27	1.986631	0.01079	0.503365	0.245075
ERG	26	2.008021	0.008387	0.498003	0.265101
KDM5B	26	1.986631	0.008951	0.503365	0.259557
CTCF	25	2.034759	0.009876	0.491459	0.25205
MYC	25	2.013369	0.008083	0.49668	0.27092
RUNX1	24	2.034759	0.006933	0.491459	0.277477
SPI1	23	2.072193	0.00707	0.482581	0.250994
ZNF143	22	2.066845	0.00628	0.483829	0.255913
MAZ	22	2.050802	0.006421	0.487614	0.279362
ELF1	22	2.05615	0.005904	0.486346	0.298782
ARNTL	22	2.109626	0.005538	0.474018	0.27185
SP1	22	2.061497	0.007389	0.485084	0.278977
TCF3	21	2.088235	0.005238	0.478873	0.281495
PHF8	21	2.136364	0.004093	0.468085	0.295021
CEBPB	21	2.125668	0.006218	0.47044	0.272461
TCF12	21	2.114973	0.005147	0.472819	0.289542
TFAP2C	21	2.136364	0.006262	0.468085	0.266791
E2F1	20	2.040107	0.006168	0.49017	0.295552
TAF1	20	2.141711	0.004164	0.466916	0.29772
CTCFL	20	2.131016	0.004453	0.46926	0.301133
MED1	19	2.195187	0.003279	0.455542	0.301484
JUND	19	2.18984	0.005712	0.456654	0.264742
NOTCH1	19	2.088235	0.004576	0.478873	0.309831
KDM2B	19	2.147059	0.003495	0.465753	0.310989
LARP7	19	2.104278	0.004425	0.475222	0.316458
STAT1	19	2.125668	0.004486	0.47044	0.303774
E2F6	19	2.088235	0.00484	0.478873	0.274578
GATA3	19	2.163102	0.004673	0.462299	0.286357
TRIM28	19	2.147059	0.004839	0.465753	0.297788
The top 30 TFs with the highest degree in DEmiRNA-TF network of BMSC osteodifferentiation					
Name	Degree	Average shortest path length	Betweenness centrality	Closeness centrality	Topological coefficient
MAX	20	2.021505	0.003652	0.494681	0.161047
AR	20	2.010753	0.010422	0.497326	0.149037
MYC	18	2.032258	0.002722	0.492063	0.175405
ESR1	18	2.02509	0.004109	0.493805	0.154739
MAZ	17	2.050179	0.003885	0.487762	0.163923
FOXA1	17	2.057348	0.004905	0.486063	0.139836
ERG	17	2.039427	0.002605	0.490334	0.182422
HIF1A	16	2.035842	0.00274	0.491197	0.186531
CREB1	16	2.046595	0.003777	0.488616	0.172636
EP300	15	2.050179	0.00182	0.487762	0.20078
CTCF	15	2.043011	0.002819	0.489474	0.177864
FLI1	14	2.057348	0.001999	0.486063	0.19308
BRD4	14	2.050179	0.001697	0.487762	0.205114
TP53	13	2.064516	0.002431	0.484375	0.200512
TFAP2C	13	2.071685	0.002276	0.482699	0.183618
TCF12	13	2.060932	0.001517	0.485217	0.214543
RUNX1	13	2.071685	0.001542	0.482699	0.210065
RAD21	13	2.0681	0.002309	0.483536	0.174057
KDM5B	13	2.057348	0.001707	0.486063	0.211276
CEBPB	13	2.071685	0.003446	0.482699	0.156718
TRIM28	12	2.0681	0.001403	0.483536	0.222766
TEAD4	12	2.064516	0.001834	0.484375	0.212077
STAT1	12	2.0681	0.001237	0.483536	0.229126
SPI1	12	2.075269	0.004133	0.481865	0.206451
PHF8	12	2.071685	0.001465	0.482699	0.222712
E2F1	12	2.0681	0.001526	0.483536	0.215917
TCF3	11	2.082437	0.001244	0.480207	0.225841
REST	11	2.057348	0.00601	0.486063	0.207061
NFE2	11	2.071685	0.00123	0.482699	0.231276
MYCN	11	2.071685	0.001787	0.482699	0.231098
LARP7	11	2.082437	0.001129	0.480207	0.235147
KDM2B	11	2.075269	0.00107	0.481865	0.23975
HEY1	11	2.078853	0.001289	0.481034	0.231113
ELF1	11	2.089606	0.001158	0.478559	0.227812
EBF1	11	2.075269	0.001284	0.481865	0.220856
ARNTL	11	2.082437	0.001177	0.480207	0.22781

**Table 5:** The 13 overlapping DEmiRNA-small molecular drug target interaction pairs between the DEmiRNA-small molecular interaction networks of DPSC and BMSC osteodifferentiation.

DEmiRNAs dysregulated in both DPSC and BMSC osteodifferentiation	Small molecular targets
hsa-miR-143-3p	Docosahexaenoic acid
hsa-miR-146b-5p	5-fluorouracil
	Arsenic trioxide
	Atorvastatin
	Progesterone
hsa-miR-34c-5p	Arsenic trioxide
	Curcumin
	Glucose
hsa-miR-671-5p	5-fluorouracil
	Bromocriptine
	Microcystin-LR (MC-LR)
	Narangin
	Proanthocyanin

**Table 6:** The targeting relationship between 19 overlapping small molecule drugs and their regulated DEmiRNAs, respectively, expressed in DPSC and BMSC osteodifferentiation process. These 19 overlapping small molecular drugs can not only regulate the DEmiRNAs dysregulated in DPSC osteodifferentiation but also regulate the DEmiRNAs dysregulated in BMSC osteodifferentiation.

Small molecule	Regulated DEmiRNAs involved in DPSC osteodifferentiation	Regulated DEmiRNAs involved in BMSC osteodifferentiation
5-fluorouracil	hsa-miR-1246	hsa-miR-140-3p
	hsa-miR-146b-5p	hsa-miR-146b-5p
	hsa-miR-184	hsa-miR-342-3p
	hsa-miR-210	hsa-miR-3658
	hsa-miR-4791	hsa-miR-378i
	hsa-miR-671-5p	hsa-miR-423-5p
		hsa-miR-574-3p
		hsa-miR-671-5p
Anthocyanin	hsa-miR-335-5p	hsa-miR-450a-5p
Arsenic trioxide	hsa-miR-133b	hsa-miR-146b-5p
	hsa-miR-146b-5p	hsa-miR-34c-5p
	hsa-miR-184	
	hsa-miR-210	
	hsa-miR-34c-5p	
Ascorbate	hsa-miR-1246	hsa-miR-1972
	hsa-miR-134	
	hsa-miR-1973	
Atorvastatin	hsa-miR-146b-5p	hsa-miR-146b-5p
	hsa-miR-487a	hsa-miR-224-5p
		hsa-miR-548d-5p
Bromocriptine	hsa-miR-671-5p	hsa-miR-671-5p
Curcumin	hsa-miR-210	hsa-miR-34c-5p
	hsa-miR-335-5p	hsa-miR-450a-5p
	hsa-miR-34c-5p	
Docosahexaenoic acid	hsa-miR-1283	hsa-miR-141-3p
	hsa-miR-143-3p	hsa-miR-143-3p
	hsa-miR-181a-5p	hsa-miR-191-5p
		hsa-miR-193b-3p
Ginsenoside Rh2	hsa-miR-210	hsa-miR-188-5p
	hsa-miR-3195	hsa-miR-483-3p
	hsa-miR-3656	hsa-miR-630
	hsa-miR-370	
	hsa-miR-4284	
Glucose	hsa-miR-133a	hsa-miR-129-5p
	hsa-miR-133b	hsa-miR-199b-5p
	hsa-miR-329	hsa-miR-342-5p
	hsa-miR-34c-5p	hsa-miR-34c-5p
	hsa-miR-615-3p	hsa-miR-369-3p
		hsa-miR-508-3p
		hsa-miR-520b
		hsa-miR-525-5p
		hsa-miR-548d-5p
Hesperidin	hsa-miR-133b	hsa-miR-188-5p
		hsa-miR-450b-3p
Hydroxycamptothecin (HCPT)	hsa-miR-1246	hsa-miR-10a-5p
	hsa-miR-1973	hsa-miR-135a-3p
	hsa-miR-335-3p	hsa-miR-181a-2-3p
	hsa-miR-370	hsa-miR-1972
	hsa-miR-543	hsa-miR-224-3p
Microcystin-LR (MC-LR)	hsa-miR-671-5p	hsa-miR-671-5p
Mistletoe lectin-I	hsa-miR-331-3p	hsa-miR-369-3p
	hsa-miR-615-3p	hsa-miR-491-3p
Narangin	hsa-miR-671-5p	hsa-miR-188-5p
		hsa-miR-671-5p
Proanthocyanin	hsa-miR-133a	hsa-miR-671-5p
	hsa-miR-133b	
	hsa-miR-671-5p	
Progesterone	hsa-miR-146b-5p	hsa-miR-146b-5p
	hsa-miR-370	hsa-miR-525-5p
Vitamin D3	hsa-miR-133b	hsa-miR-339-5p
	hsa-miR-331-3p	
	hsa-miR-543	
Vorinostat (SAHA)	hsa-miR-134	hsa-miR-542-3p
	hsa-miR-409-3p	hsa-miR-574-3p

## Data Availability

The data used to support the findings of this study are available from the corresponding author upon reasonable request.

## Supplementary Materials

Supplementary 1 File S1 The DEmiRNAs dysregulated in the osteodifferentiation of DPSC.

Supplementary 2 File S2 The DEmiRNAs dysregulated in the osteodifferentiation of BMSC.

Supplementary 3 File S3 The topological characteristics of all nodes in the 16 shared DEmiRNAs-target gene network.

Supplementary 4 File S4 The topological characteristics of all nodes in the DEmiRNAs-transcription factor interaction network of DPSCs osteodifferentiation.

Supplementary 5 File S5 The topological characteristics of all nodes in the DEmiRNAs-transcription factor interaction network of BMSCs osteodifferentiation.
